The article "Do Gender or Major Influence the Performance in Programming Learning? Teaching Mode Decision Based on Exercise Series Analysis" was published in 2022. Journal: Comput Intell Neurosci.

# Do Gender or Major Influence the Performance in Programming Learning? Teaching Mode Decision Based on Exercise Series Analysis

**DOI:** 10.1155/2022/7450669

**Published:** 2022-02-08

**Authors:** Zhizezhang Gao, Yan Zhang, RuiPeng Zhang, Xia Sun, Jun Feng

**Affiliations:** Northwest University, Xi'an, ShaanXi, China

## Abstract

Both traditional teaching and online teaching advocate individualized education. One of the difficulties on exploring possible improvements of instructional design is the challenging process of data collection. Existing research mainly focuses on the exam score of students but pays little attention to students' daily practice. As an effective method to handle time-series dataset, the generalized estimating equations (GEE) have not been used in this research field. Considering above issues, we first propose an experimental paradigm of programming performance analysis based on the performance record of students' daily practice-exam and finish collecting a complete time-series dataset in one semester, including students' individual attributes, learning behavior, and learning performance. Then, we propose an approach that analyzes practice-exam time-series dataset based on GEE to study the influence of individual attributes and learning behavior on learning performance. It is the first time to apply the GEE method for ordinal multinomial responses in this research field, by which we conclude several results that gender or major does have a certain difference on the programming learning. The longer the answer time and the less the cost time, the better the students' performance. Regardless of gender, students tend to cram for the exam and perform a little worse in the daily exercise. Finally, targeting at two important individual attributes, we give corresponding teaching mode decisions that university should teach students programming by major and teacher should give different teaching methods to students of different genders at different time points.

## 1. Introduction

The last decade has witnessed an explosion in the number of web-based education systems due to the increasing demand in higher-level education [1], limited number of teaching personnel, and advances in information technology and artificial intelligence. However, there are significant limitations of currently available online teaching platforms. Since courses are taken online, there is no interaction between the students and the teacher as in a classroom setting, which makes it difficult to meet the personalized needs of each student.

In order to meet the needs of personalized teaching, researchers have conducted a lot of research on the factors that affect students' academic performance. The influencing factors mainly included students' personal characteristics and learning behaviors [2].

Researchers suppose that personal characteristics predispose academic performance. Differences in these characteristics cause individuals to react to learning in their own ways [3]. Many researchers also underpinned the importance of individual differences in personal characteristics for learning outcome [4–6]. Learners had ideas and beliefs with regard to learning and these learning conceptions are essential for the development of learning activities [7, 8]. Motivational orientations as well as regulation strategies had proven to be significant in students' learning processes [9]. In 2007, Van Bragt showed that learning conceptions, learning orientations and regulation strategies were not separated concepts, but rather different aspects of one concept referring to “personal orientations on learning” [10]. The quality of learning processes and study outcome was assumed to be heavily dependent on the quality of students' study approach [11]. An indirect relationship existed between conceptions and achievement as well as dropout, mediated by actual learning activities [12].

By conducting descriptive statistical analysis in comparing two different courses in MOOC platform, Shukor and Abdullah's research suggested that using learning analytics in MOOC could help enhance the instructional design, thus improving the learning retention and engagement [13]. Focusing on quality assurance of language courses, Luo and Ye examined what has influenced learners' perceptions and identifies the specific quality criteria of five types of them with the data collected from English as a second language learners on China's biggest MOOC platform “iCourse” through qualitative study [14].

Other studies focused on student learning behavior. In 2006, Bernhard et al. combined a standardized diary approach with time-series analysis methods to investigate the process of self-regulated learning, and the result of trend analyses demonstrated the effectiveness of the intervention, which consists of four weekly training sessions and had significant improvements in self-regulatory behavior [15].

Gillani studied a particular course in Coursera with the datasets of nearly 87000 students' learning behavior and achievement using social network analysis, and the result showed that those who engage explicitly in the discussion forums are more likely to have better performance than their counterparts in the course, although the vast majority of forum participants receive “failing” marks [16].

In 2014, Jia et al. collected 82352 students' learning behavior of six courses released by Peking university in Coursera and explored their influence on students' achievement by correlation analysis, the result showed that the score of common tests and the activity level in the forum have a strong positive correlation with final achievement in the course, and the number of visiting course web pages had a certain positive influence on the final achievement [17].

In 2015, Li et al. used a Tobit and Logit model to analyze factors of learning behavior that influenced the participation, completion, and achievement in the course, and they found that students with stronger learning motivation have higher course participation, earlier registered in the course, more active participation, and better completion and achievement [18]. Based on the same dataset, Jiang et al. classified students into several groups by the characteristics of learning behavior and used three classification models to deeply explore the relationship between learning behavior and learning achievement [19].

In 2017, Su et al. proposed a big data analysis technique on learning portfolio to explore how the interaction, unknown correlations, and hidden patterns among learners on MOOCs and social media platforms start and recognize the using big data analytics transforming on students' learning behavior [20]. Martina et al. analyzed data from users of an online platform that provides learning materials for medical students in preparation for their final exams and found correlations between the number of cards studied and the number of test questions that had been answered with the percentage of correct answers in the learners' medical exams through hierarchical regression analysis [21].

In 2017, Sanghoon got a finding of a comparative analysis of online learner behavioral interactions, time-on-task, attendance, and performance at different points throughout a semester based on two online courses: one course offering authentic discussion-based learning activities and the other course offering authentic design/development-based learning activities through a series of Mann–Whitney tests, and the result indicates that at the beginning of the semester, students who were involved in authentic design/development-based learning activities showed a significantly higher number of behavioral interactions with the Moodle LMS than those who involved in authentic discussion-based learning activities. However, students who were given authentic design/development-based learning activities received higher performance scores both during the semester and at the end of the semester [22].

Based on the research on online learning behavior in 2019, Cai proposed an online learning behavior analysis strategy design that promotes online course learning. Cai selected 30 learners to conduct specific learning experiments to verify the impact of learning analysis on curriculum learning. According to the evaluation results of learning effect, online learning analysis can achieve good learning results, which is helpful for students to improve their learning effect and teachers to improve teaching effect, and can be better applied to the teaching practice of online course [23].

In 2019, Rong et al. developed MPT discrete values of the time-series model based on the traditional first-order mixed Thinning and Pegram operators into a new higher-order MPT(p) model, and they first studied the autocorrelation structure and analyzed the methods of model order and parameter estimation, and then deduced the properties of parameters and regression as well as presented the prediction method of the model. Finally, by modeling the discrete data sequence of the MOOC course's learning behavior, they described online learners' behavior characteristics and discovered the dependent influence of higher-order delay of online learning behavior, realizing the short-term prediction of discrete sequence [24].

In 2021, Spitzer et al. have investigated students' engagement with the online learning environment Bettermarks for mathematics by using survival analysis. Particularly, this research was done during the COVID-19 pandemic era. The study revealed that the total number of students using the online learning environment increased significantly during and after school closure, while students' engagement decreased faster over time [25].

In 2021, Huang et al. analyzed online learning behavior data from the “Moso Education” cloud platform through correlation analysis, cluster analysis, and analytic hierarchy process analysis. They found that problem-solving behavior of learners is of the least importance, which is not common in online learning behavior, while social interaction behavior is better than problem-solving behavior, and resource learning behavior is the most common in online learning. The score distribution diagram of resource learning behavior shows an inverse s-shaped curve, while the curves of the score distribution diagram of social interaction behavior and problem-solving behavior are close to a straight line. There are learning achievement differences in resource learning behavior and problem-solving behavior, and core-marginal differences in resource learning behavior and social interaction behavior [26].

In the above studies, the use of static behavior attributes accounted for the majority, and the models used in the field of time series are few and simple. This is based on the presence of difficulties in collecting dynamic behavior attributes. This paper uses a GEE model that has not been widely used in the education field. Previously, it was mainly used in the medical and social research fields to model and analyze time-series data or repeated measurement data [27].

At the same time, the dataset used in this article is a semester-related time-series dataset in the programming course, and it distinguishes between exercise and test data—this is due to the big difference in time series between exercises and the test.

Considering above issues, we aim to analyze the influence of students' personal attributes and learning behavior on learning performance in programming to help improve scaffolding instructional design of courses in university by the generalized estimating equations (GEE) method for ordinal multinomial responses in *R*, with elaborated design and collection of time-series dataset from the PTA platform. We summarize our key contributions as follows:

1. We propose a course performance analysis experimental paradigm based on practice-test assessment records and collect a semester-related time-series dataset to provide a basis for high-quality scientific monitoring of students' academic performance process modeling
2. We proposed a GEE-based practice-test time-series analysis method and mined attribute factors related to academic performance
3. We put forward corresponding teaching method decisions for important related factors

## 2. Materials and Methods

### 2.1. Experimental Setup

According to characteristics of programming, we elaborately select five types of question in each exercise: true-false test, multiple-choice test, cloze of programming, writing function, and programming. Exercise is organized and released by teachers every week regularly, among them the exercise series are divided into two parts: practice series and exam series. The difference between them is that students must finish the exam exercise under the supervision of teacher in special classroom within 2 hours including midterm exam and final exam, while the practice could be finished anywhere and anytime without supervision during the limited time set by teachers which is usually a week, so students could have more time to review knowledge and finish practice. During the process of practice and exam, their learning behaviors (e.g., answer time and cost time) and learning performance (scores of each exercise and exam) are recorded. Students' learning behavior is time-varying.

We choose an experimental class of Northwest university as case study including 75 students of different genders, majors, and basis in the first year of college. They enroll in a compulsory course, Programming, during a 4-month semester. The course uses a face-to-face teaching method, which ensures that each student receives the same teaching process from the course. At the first class, each student is asked to participate in a questionnaire including the information of personal attributes (e.g., their genders, majors, and basis). In total, there are 50 men and 25 females, 35 students major in mathematics and 40 students major in computer science, and 30 students who have learnt about computer programming systematically before the course (actually before entering university because they are the freshmen in university). Students' individual attributes are constant and do not change over time.

### 2.2. Data Collection and Dataset Construction

The data collection is completed through an online exercise platform called PTA (https://pintia.cn), which was designed and developed by Zhejiang University in China targeting at the online exercise in programming. Each time when students make their exercise or exam, their learning behaviors and learning performance are recorded in the PTA platform. So, we could obtain a complete exercise-series dataset from the PTA platform. The dataset consists of exam samples and practice samples. The exam samples are two-stage time-series data from midterm exam to final exam, containing 150 observations. The practice samples consist of 13 exercises during the whole course, containing 1044 observations.

The meaning of variables used in this research is described as follows:

1. Learning performance, collected from PTA platform: while score measures the students' learning performance in each exercise and exam which all have a total score of 100 points, considering the different knowledge points and difficulty or extent examined in each exam or exercise, we standardized each score by the mean and standard deviation of its contemporaneous exercise to give a relatively objective and fair evaluation about learning effect of each student. And we make score after standardization less than −1 as “poor,” greater than −1 less than 1 as “medium,” and greater than 1 as “excellent,” which are assigned to the value of 1, 2, and 3, respectively.
2. Gender, individual attribute collected from questionnaire at the first class: We assign men to 1 and female to 2.
3. Major, individual attribute collected from questionnaire at the first class: this experimental class has two types of major, mathematics and computer science, of which there are 35 students major in mathematics and 40 students major in computer science. We assign mathematics to 1 and computer science to 2.
4. Basis, individual attribute collected from questionnaire at the first class: this variable reflects whether a student has learned about computer programming systematically before the class, their answers are “Yes” or “No,” of which we assign “No” to 1, and “Yes” to 2.

Sequence of exercise, as the time variable, this variable is the sequence of score in exercise series collected in the PTA platform. In exam samples, its value are 1 and 2, which represent midterm exam and final exam. In practice samples, its value ranges from 1 to 13, which represent the thirteen exercises during the whole course.

Answer time, learning behavior collected in the PTA platform: This variable measures the time that a student costs in finishing one exercise. The unit is second resulting in the large value range. To linearize this variable and reduce heteroscedasticity, we process the answer time with logarithm. This variable partly reflects the degree of effort on exercise and the degree of mastery on knowledge. From our teaching practice, longer answer time usually means that more seriousness and effort are given to exercise resulting in better performance, which is still required to be proved by data analysis.

Cost time, learning behavior collected in the PTA platform: This variable measures the time difference from the time teacher releases the exercise on PTA platform to the time student finishes it. The unit is second too. So we also process the cost time with logarithm. This variable partly reflects the degree of enthusiasm on studying. According to our teaching practice, longer cost time usually means that students tend to be more dilatory and more likely to finish exercise hastily before the deadline even copy the other's answer, which we think may result in worse performance and needs further data analysis to confirm.

Variables of exam samples include learning performance, gender, major, basis, and sequence without answer time or cost time because the exam is held with limited time and most students do not end up answering until the time of exam is over. Practice samples include all variables mentioned above: gender, major, basis, and sequence. And these four variables do not change over time, and nevertheless, three variables of learning performance, answer time, and cost time change over time.

The definitions and value setting of above variables are summarized in Table 1:

### 2.3. Exercise Series Analysis Based on GEE

Considering that the datasets actually both are time-series data (or called repeated measured data, longitudinal data), we propose an approach to analyze practice-exam time-series dataset based on GEE to study the influence of individual attributes and learning behavior on learning performance, which has been proved to be an effective method on handling time-series dataset but has not been used in this research field.

Liang and Zeger [28] originally proposed the GEE method as an extension of generalized linear models to handle longitudinal data. The biggest advantage of the GEE is that we do not need to specify the whole distribution of the response. Only the mean structure and the mean-variance relationship and specification of the covariance structure need to be defined [29].

Let (*y*_*it*_, *x*_*it*_) be observation data, *i*=1,…, *n*; *t*=1,…, *T*_*i*_, and expected value and variance of measurement *y*_*it*_ can be expressed using a generalized linear model:

(1) $$\begin{array}{c} \mu_{it}=E\left(y_{it}\right)=g^{-1}\left(x_{it}^{T}\beta \right);\\ \text{Var}\left(y_{it}\right)=\phi V\left(\mu_{it}\right). \end{array}$$

where *g* is a link function with known form, *V* is a variance function with known form, *β* is an unknown vector of regression coefficients, and *ϕ* is a scale parameter.

The parameters *β* are estimated by solving: $U\left(\beta ,\hat{\alpha }\right)=\sum_{i=1}^{n}\partial \mu_{i}/\partial \beta \;V_{i}{\left(\alpha \right)}^{-1}\left(y_{i}-\mu_{i}\right)=0$, where *y*_*i*_=(*y*_*i*1_, *y*_*i*2_,…,*y*_*iT*_*i*__)^*T*^, *μ*_*i*_=(*μ*_*i*1_, *μ*_*i*2_,…,*μ*_*iT*_*i*__)^*T*^, and *α* denotes a vector of association parameters. The variance-covariance matrix for *y*_*i*_ is noted by *V*_*i*_(*α*)=*A*_*i*_^1/2^*R*_*i*_(*α*)*A*_*i*_^1/2^*A*_*i*_=diag{v(*μ*_*i*1_),…, v(*μ*_*iT*_*i*__)}, and the so-called “working correlation structure” *R*_*i*_(*α*) describes the pattern of measures within the subjects, which has 4 following options:

1. Independent: it is uncorrelated between any two time points
2. Exchangeable: consider all correlations equal
3. Autoregressive: there is a correlation dependent on the time between measurements
4. Unstructured: no form of correlation is specified in advance

In 2013, Anestis et al. propose a GEE approach for correlated ordinal or nominal multinomial responses using a local odds ratios parameterization [30]. They treat *α* as a “nuisance” parameter vector that defines the local odds ratios structure at the marginalized contingency tables after tabulating the responses without a covariate adjustment at each time pair. There are also 4 options for the association model:

1. Uniform structure: assume exchangeability of time pairs and of adjacent-category pairs
2. Category exchangeability structure: assume a common local odds ratio at each time pair, but permits different pairs to have differing associations
3. Time exchangeability structure: this structure does not assume any time dependency and it implies equal local odds ratios at different category cutpoints
4. RC structure: an extension of the previous structure that additionally allows a time dependency

In 2015, Anestis offers an *R* package multgee for modeling ordinal or nominal multinomial responses in *R* [27], which is used to process and model data in this paper.

We focus on modeling the influence of students' individual attributes and learning behavior on learning performance. Considering that the value of processed learning performance is “poor,” “medium,” and “excellent” from bad to good, so we set learning performance as an ordinal multinomial variable and it is the dependent variable *Y*. Because gender, major, and basis are categorical variables, so we make them as nominal or multinomial variables by introducing dummy variables in the GEE model. Processing answer time and cost time with logarithm before, we make them as numeric variables with answer time abbreviated to “AT” and cost time abbreviated to “CT” in the GEE model. Using “time” to express sequence intuitively in the model, we set time as nominal variable when we model exam samples. With regard to practice samples, when we examine the overall tendency of change in students' learning performance series and the cross effect between time and the other variables, we set time as numeric variable. When we examine the process of change among students' learning performance series, we set time as nominal variable. The range of the estimated intrinsic parameters is big (14.35–(−0.46) = 14.81), which suggests that the underlying association pattern exists across time-pairs, so we choose time exchangeability structure as a model structure in our research.

Take exam samples for example, the marginal cumulative logit model based on GEE

(2) $$\begin{array}{c} \text{log}\left(\frac{P\left(Y_{i\text{t}}\leq j\right)}{1-P\left(Y_{i\text{t}}\leq j\right)}\right)=\beta_{0j}-\beta_{1}I\left\{{\text{gender}}_{i}=\text{female}\right\}-\beta_{2}I\left\{{\text{major}}_{i}=\text{computer science}\right\}-\beta_{3}I\left\{{\text{basis}}_{i}=\text{yes}\right\}\\ -\beta_{4}I\left\{\text{time}=\text{final exam}\right\}-\beta_{5}I\left\{{\text{gender}}_{i}=\text{female}\right\}\times I\left\{\text{time}=\text{final exam}\right\}\\ -\beta_{6}I\left\{{\text{major}}_{i}=\text{computer science}\right\}\times I\left\{\text{time}=\text{final exam}\right\}\\ -\beta_{7}I\left\{{\text{basis}}_{i}=\text{yes}\right\}\times I\left\{\text{time}=\text{final exam}\right\}. \end{array}$$

is fitted in this paper, where *i*=1,2,…, 75, *t*=1,2,  *j*=1,2, and *I*(*A*) is the indicator function for the event A. Gender, major, and basis are nominal variables and not time-varying, AT and CT are numeric variables and time-varying, and time is nominal variable and time-varying. *β*_1_, *β*_2_, *β*_3_, *β*_4_ measure the respective effect of gender, major, basis, and time on learning performance, and *β*_5_, *β*_6_, *β*_7_ measure the cross effect with time.

For practice samples setting time as numeric variable, the marginal cumulative logit model based on GEE

(3) $$\begin{array}{c} \text{log}\left(\frac{P\left(Y_{i\text{t}}\leq j\right)}{1-P\left(Y_{i\text{t}}\leq j\right)}\right)=\beta_{0j}-\beta_{1}I\left\{{\text{gender}}_{i}=\text{female}\right\}-\beta_{2}I\left\{{\text{major}}_{i}=\text{computer science}\right\}-\beta_{3}I\left\{{\text{basis}}_{i}=\text{Yes}\right\}\\ -\beta_{4}\text{time}-\beta_{5}AT_{it}-\beta_{6}CT_{it}-\beta_{7}I\left\{{\text{gender}}_{i}=\text{female}\right\}\times \text{time}\\ -\beta_{8}I\left\{{\text{major}}_{i}=\text{computer science}\right\}\times \text{time}-\beta_{9}I\left\{{\text{basis}}_{i}=\text{yes}\right\}\times \text{time}\\ -\beta_{10}AT_{it}\times \text{time}-\beta_{11}CT_{it}\times \text{time}. \end{array}$$

is fitted in this paper, where *i*=1,2,…, 75, *t* & time=1,2,…, 13, *j*=1,2, similar form of expression with above. And the model of practice samples setting time as nominal variable is omitted here for its tedium.

## 3. Results and Discussion

In our teaching practice, we found that major and gender may have differences on students' academic performance. Therefore, in this part, we hope to use the results of quantitative research to explore the following problems:

  RQ1: should university teach students programming by major according to the different demands?
  RQ2: should teacher give different teaching methods to students of different genders?

### 3.1. Regression Results of GEE Model

We use *R* package “multgee” to construct the marginal cumulative logit models based on GEE mentioned in Section 2.3. All the results of coefficient estimate are showed in this section. In Tables 2–7, we examine the cross term of the variables that are not time-varying and time to explore change tendency of their influence over time. Tables 5–7 are generated by setting time variable as numeric variable in the GEE model.  Figure 1 is generated by setting time variable as nominal variable in the GEE model to examine the tendency between exercises.  Table 8 is generated by setting gender as dependent variable, and answer time and cost time as independent variables to explore the relationship existed among gender, answer time, and cost time.

Table 2 shows the regression result of the whole sample of exam, we could see that computer science has a significant positive influence on learning performance of exam, and the influence of the female on learning performance has a significant negative tendency. Tables 3 and 4 show the regression result of subsample of exam in gender and major, and we could see the comparison between different majors and genders.  Table 5 shows the regression result of the whole sample of practice, we could find that computer science also has a significant positive influence on learning performance of practice, and students' performance is improving over time. The teaching experience about the influence of answer time and cost time mentioned in Section 2.2 is confirmed by the quantitative analysis. Tables 6 and 7 show the regression result of subsample of practice in gender and major; in Table 6, we found that the influence brought by a major difference is bigger in men than in females, and students major in computer science perform much better than mathematics. In Table 7, we find that gender differences have a greater impact on computer science than on mathematics, and the two effects are in the opposite direction. Among them, females majoring in mathematics are better than men, while men majoring in computer science are significantly better than women.  Table 8 shows the regression result by setting gender as dependent variable, and answer time and cost time as independent variables; it could be concluded that females tend to have longer answer time and cost time.  Figure 1 shows the trend of students' relevant performance in exercise compared with the first exercise.

About the exact meaning of coefficient estimate, for instance, the estimate of computer science in Table 2 suggests that cumulative probability (*P*(*Y*_*i*t_ ≤ *j*)) starting at the well end of the scale increases when students' major is computer science not mathematics. Given a fixed learning performance, at the “computer science,” the estimated odds of learning performance below any fixed level are *e*^1.0326^=2.8084 times the estimated odds at the “mathematics.”

About the exact meaning of coefficient estimate, for instance, the estimate of computer science in Table 2 suggests that cumulative probability (*P*(*Y*_*i*t_ ≤ *j*)) starting at the well end of the scale increases when students' major is computer science not mathematics. Given a fixed learning performance, at the “computer science” the estimated odds of learning performance below any fixed level are *e*^1.0326^=2.8084 times the estimated odds at the “mathematics.”

### 3.2. Discussion and Teaching Model Decision

From Table 2, we found that compared with the students' major in mathematics, the students' major in computer science significantly has a higher level of score in the exam, and this positive influence tends to decrease over time, which means that for the learning in the programming class under the same teacher and environment, students major in computer give more effort to this course than students major in mathematics, while all students are freshmen in the university. The reason we think is that programming is the foundation of other future classes or the skill lived by for students major in computer, so it results in more attention given to this course, and students major in mathematics has to take effort finally forced by the pressure of score. And a female performs a certain better trend in the exam than a man, but this influence falls a lot significantly over time resulting in the worse performance in the final exam. In the consideration of the difficulty gradually improved during the whole course, it seems like that male tends to be more adaptable and interested in the latter period of programming class. What's more, having basis of computer is certain more helpful to the score, and this influence also falls a lot over time, so having basis will result in a certain advantage on score, but this advantage will be diluted by time or the effort in studying. Finally, students performed a little better in the final exam than the midterm exam, we think that students need time to gradually fit the study style and they have to pay more attention and effort to study before the final exam forced by the pressure of score.

Table 3 shows the experiment results in two subsamples of gender, from which we could see that major and basis differences have greater positive impacts on the score of a female, and these impacts tend to decline more than they do on the score of a male over time. And men performed better over time, while females even performed a little worse over time. So, the influence brought by the difference of major and basis mentioned in Table 2 is much bigger in females than in men, and this influence will be diluted over time.

We found in Table 4 that gender and basis differences have a greater positive influence on the score of students' major in mathematics than in computer science. And the positive influence of gender difference falls a lot over time, of which the decrease is larger in computer science than in mathematics. The time-varying tendency differs in basis, and the positive influence brought by a basis difference falls a lot in mathematics and increases little in computer science.

In Table 5, we could see that students major in computer science performs significantly better in the exercises than students major in mathematics, and this influence remains largely the same over time. Females tend to have a lower score than men, which is significantly improved over time. Having basis or not does not have so much difference on the influence in score or change over time. As a whole, students' performance is improving over time. The answer time longer and the cost time shorter, the score of exercise will be higher. We think that the answer time longer, more seriously students finish the exercise, and the cost time shorter, students tend to treat the exercise more actively and to be less dilatory, so it is not strange to see the score, which tends to be improved.

From Figure 1, we can see that the performance of students improves significantly in the exercise before the midterm exam and the final exam, and a little worse in other daily exercise. What's more, females perform better than men. So, we conclude that students did not pay enough effort to the exercise until exams, and females tend to be more diligent than men. So, it seems that students all like to cram for the exam.

Combining the above results of exam sample and practice sample, we could conclude that for RQ1 university had better teach students programming by major because students' learning performance in exam and practice shows a significant difference on major, or teachers should add some content related to their major in teaching to drag interest of students not major in computer science and improve their subjective initiative or degree of attention, and urge them more to study at the same time. And among students major in computer science, teachers should pay more attention to the learning of females because the gender difference is significantly enlarged over time.

For RQ2, teachers should give different teaching methods to students of different genders. More attention should be given to females in the second half of semester for their large and significant decline on the learning performance over time maybe because of the gradually improving difficulty in programming. And men prefer to challenge the improving difficulty and actually perform better than females. But teachers should urge men more for their relative low learning performance in exercise, and females seem to be more conscious and diligent than men in daily practice. And this phenomenon is also likely to be consistent with the characteristics of programming.

## 4. Conclusion

In this paper, we propose a new experimental paradigm in studying the students' performance in programming learning. Based on the elaborately collected exercise-series dataset, our research focus on not only the final exam result but also daily performance to explore what roles gender and major play in the process of programming learning, according to which we give our recommended decisions on programming teaching model in university. But until now, we only know what happened by the regression result, and we still do not know exactly why the influence happened. So, this is our future research direction to study more.

## Figures and Tables

**Figure 1:** Students' relevant performance of exercise compared with the first exercise.

**Table 1:** Definitions and value settings of variables used in this research.

Variable	Definition	Value
Learning performance	It measures the students' learning performance, standardized by the mean and standard deviation. Less than −1 as “poor,” greater than −1, less than 1 as “medium,” and greater than 1 as “excellent”	Poor = 1
		Medium = 2
		Excellent = 3
Gender	Sex of students in this class, male or female	Male = 1; female = 2
Major	Student's major, mathematics or computer science	Mathematics = 1
		Computer science = 2
Basis	Whether a student has learned about computer programming systematically before the class: no or yes	No = 1; Yes = 2
Sequence	Sequence of each score in exam or exercise	Exam samples: 1, 2
		Practice samples: From 1 to 13
Answer time	The time that a student cost in one exercise	Process answer time with logarithm
Cost time	The time difference from the time teacher releases the exercise on PTA platform to the time student finishes it	Process cost time with logarithm

**Table 2:** Regression result of the whole sample of exam.

Variable	Coefficient estimate
Mathematics	
Computer science	1.0326^*∗*^
Man	
Female	0.1569
Time = Midterm exam	
Time = Final exam	0.8198
Basis = No	
Basis = Yes	0.7958
Computer science × time	−0.2970
Woman × time	−1.0011^*∗*^
Basis=Yes × time	−0.6788

^*∗*^Significance at 0.10, ^*∗∗*^significance at 0.05, ^*∗∗∗*^significance at 0.01, which is similar in all tables.

**Table 3:** Regression result of subsample of exam in gender.

Variable	Coefficients' estimate of male sample	Coefficients estimate of female sample
Mathematics		
Computer science	0.9068	1.5524
Time = midterm exam		
Time = final exam	0.6109	−0.0604
Basis = no		
Basis = yes	0.6256	1.5100
Computer science × time	−0.1823	−0.7391
Basis=yes × time	−0.4997	−1.3576

**Table 4:** Regression result of subsample of exam in major.

Variable	Coefficients' estimate of mathematics sample	Coefficients' estimate of computer science sample
Man		
Female	0.2509	0.0676
Time = midterm exam		
Time = final exam	1.1116	0.0028
Basis = No		
Basis = yes	1.4125^*∗∗*^	0.1248
Woman × time	−0.9216	−1.1848^*∗*^
Basis=yes × time	−1.3591	0.0736

**Table 5:** Regression result of the whole sample of practice.

Variable	Coefficient estimate
Mathematics	
Computer science	0.4437^*∗∗*^
Man	
Female	−0.3424
Basis = no	
Basis = yes	0.0450
Time	1.1515^*∗∗∗*^
Answer time	4.2368^*∗∗∗*^
Cost time	−0.0519
Basis=yes × time	0.0369
woman × time	0.0551^*∗∗*^
Computer science × time	−0.0209
Answer time × time	−0.3683^*∗∗∗*^
Cost time × time	0.0394

**Table 6:** Regression result of subsample of practice in gender.

Variable	Coefficients' estimate of male sample	Coefficients' estimate of female sample
Mathematics		
Computer science	0.7939^*∗∗∗*^	−0.1290
Basis = no		
Basis = yes	0.1713	−0.3320
Time	−0.0330	−0.0647^*∗*^
Answer time	0.8062^*∗∗∗*^	0.7116^*∗∗∗*^
Cost time	0.3093^*∗∗∗*^	0.4154^*∗∗∗*^
Basis=yes × time	−0.0139	0.1023^*∗∗∗*^
Computer science × time	−0.0441	−0.0110

**Table 7:** Regression result of subsample of practice in major.

Variable	Coefficients' estimate of mathematics sample	Coefficients' estimate of computer science sample
Man		
Female	0.1740	−0.9538^*∗∗∗*^
Basis = no		
Basis = yes	0.1721	−0.1110
Time	−0.0766^*∗∗*^	−0.0876^*∗∗∗*^
Answer time	0.8608^*∗∗∗*^	0.6529^*∗∗∗*^
Cost time	0.4504^*∗∗∗*^	0.3038^*∗∗∗*^
Basis=yes × time	0.0458	0.0171
Woman × time	0.0312	0.0747^*∗∗*^

**Table 8:** Regression result by setting gender as dependent variable, and answer time and cost time as independent variables.

Variable	Coefficients estimate
Answer time	0.0713
Cost time	0.0995

## Data Availability

The dataset can be accessed via fengjun@nwu.edu.cn and sign an agreement.
